The article "miR-34 inhibits growth and promotes apoptosis of osteosarcoma in nude mice through targetly regulating TGIF2 expression" was retracted in 2024. Reason: duplicated images.

# *miR-34* inhibits growth and promotes apoptosis of osteosarcoma in nude mice through targetly regulating TGIF2 expression

**DOI:** 10.1042/BSR20180078

**Published:** 2018-06-12

**Authors:** Liang Xi, Yongfeng Zhang, Shengnan Kong, Wei Liang

**Affiliations:** 1 Department of Orthopaedic Surgery, Xijing Hospital, The Fourth Military Medical University, Xi’an 710032, China; 2 Department of Medical Oncology, Xijing Hospital, The Fourth Military Medical University, Xi’an 710032, China

**Keywords:** apoptosis, miR-34, Osteosarcoma, TGIF2, tumor volume

## Abstract

*miR-34* was reported to be involved in multiple tumors occurrence and development. The aim of the present study was to explore the impact of *miR-34* on osteosarcoma and related mechanisms. Tumor tissues and non-tumor tissues of 34 patients with osteosarcoma were collected. qRT-PCR detection revealed that *miR-34* was significantly down-regulated in tumor tissues (*P*<0.05). hFOB 1.19 and MG-63 cells were cultured. qRT-PCR detection showed that *miR-34* was also significantly down-regulated in MG-63 cells (*P*<0.05). After transfection by *miR-34* mimics, MG-63 cells proliferation in nude mice was significantly impaired (*P*<0.05), and percentage of apoptosis as well as caspase-3 positive cells proportion of osteosarcoma tissue in nude mice was markly increased (*P*<0.05). Western blot and immunofluorescence results also demonstrated that TGIF2 relative expression and TGIF2 positive cells proportion were both dramatically decreased (*P*<0.05). By luciferase reporter assay, we found that *TGIF2* was the target gene of *miR-34.* After transfected by TGIF2 overexpression vector or co-transfected by *miR-34* mimics and TGIF2 overexpression vector, we observed that, compared with blank group, tumor volume was significantly increased and apoptotic cells as well as caspase-3 positive cells proportion was obviously decreased in TGIF2 group (*P*<0.05), while no significant difference was found in these indicators between blank group and TGIF2 + mimics group. We concluded that *miR-34* inhibited growth and promoted apoptosis of osteosarcoma in nude mice through targetting regulated TGIF2 expression.

## Introduction

Osteosarcoma has a serious negative impact on bone growth and often occurs in children and adolescents [1]. It is often found in long bones and mainly occurs in the knee, with an incidence of 4.4 per million people worldwide [2]. According to reports, the 5-year survival rate is no more than 30% for osteosarcoma patients with recurrent or metastasis [3]. Over the past 30 years, improved prognosis of osteosarcoma has been achieved gradually [4]. However, the recurrence and metastasis rates remained high. Therefore, there is an urgent need to find more effective therapy method for the treatment of osteosarcoma.

Accumulated evidence showed that gene therapy could achieve a complete cure in many tumors than traditional therapies [5,6]. Abnormal expression of genes was associated with several tumors occurrence, especially miRNAs [7]. Amongst these wide varieties of miRNA, *miR-34* was reported to be associated with several tumors progress. Chamani et al. [8] thought that *miR-34* was one of the tumor suppressor miRNAs, which was expressed in majority of normal tissues. Kasinski and Slack [9] found that *miR-34* could inhibit cancer initiation and progression in mouse models of lung adenocarcinoma. Tang et al. [10] revealed that *miR-34* was a tumor suppressor gene, which could inhibit the development of human pancreatic cancer. Cheng et al. [11] demonstrated in their research that *miR-34* could co-operate with p53 in suppression of prostate cancer by joint regulation of stem cell compartment. It was also the first miRNA reported to be directly *trans*-activated by tumor suppressor p53, and it was deleted or epigenetically down-regulated in multiple cancer cell lines and human malignancies [12,13]. Many other similar studies have researched the impact of *miR-34* on tumors development. However, there are few articles researching the effect of *miR-34* on osteosarcoma biological characteristics. A major breakthrough in the treatment of osteosarcoma will be achieved if the mechanism of *miR-34* on osteosarcoma could be identified.

In the present study, the expression level of *miR-34* in osteosarcoma tumor tissues and cells was explored. The exact mechanism of *miR-34* on osteosarcoma growth and apoptosis *in vivo* by nude mice was also researched. The present study has an important guiding significance for targetted treatment of osteosarcoma at the genetic level.

## Materials and methods

### Tissue collection and cell culture

A total of 34 patients with osteosarcoma who had been diagnosed as osteosarcoma by our hospital from June 2015 to March 2017 were enrolled in the present study. These patients’ tumor tissues and non-tumor tissues were collected. Tumor tissues were obtained from sarcoma part and non-tumor tissues were collected from normal adjacent tissues from the same patients. The present study has obtained the patient’s informed consent and has been approved by Ethics Committee of First Affiliated Hospital of Fourth Military Medical University. The protocol number was QX20140916-5.

Human normal osteoblastic cell line hFOB 1.19 and human osteosarcoma cell line MG-63 were purchased from American Type Culture Collection (ATCC, U.S.A.) and were cultured in DMEM medium containing 10% fetal bovine serum (FBS) in a 5% CO_2_, 37°C, 95% humidity carbon dioxide incubator. Cells were harvested at logarithmic growth phase.

### Cells transfection

*miR-34* mimics (sense: CAAUCACUAACUCCACUGCCAU; antisense: GGCAGUGGAGUUAGUGAUUGUU), *miR-34* negtive control (sense: UUCUCCGAACGUGUCACGUTT; antisense: ACGUGACACGUUCGGAGAATT) [14], as well as TGIF2 expression vector, were purchased from RiboBio, Guangzhou, China. They were used to transfect MG-63 cells, respectively and co-transfection was also conducted by using *miR-34* mimics and TGIF2 expression vector. These transfected MG-63 cells were set as *miR-34* mimics group, NC group, TGIF2 group and TGIF2 + mimics group, respectively based on different transfection types. Transfection operation was performed by using Lipofectamine 2000 (Invitrogen, U.S.A.) according to the instructions. Cells that were successfully transfected were suspended in DMEM (containing 10% FBS) and seeded in 24-well plates at a density of 1 × 10^4^/ml for incubation. MG-63 cells without any treatment were used as blank group.

### qRT-PCR detection

Total RNA was obtained from tumor tissues and cells by using TRIzol (obtained from Invitrogen, U.S.A.). Extraction processes were strictly in accordance with the instructions. Reverse transcription reaction was used to synthesize cDNA template by using TaqMan MicroRNA Reverse Transcription Kit (bought from Applied Biosystems, U.S.A.). The sequences of the primers were as follows: *miR-34*, forward, 5′-TCTATTTGCCATCGTCTA, reverse, 5′-CAGGCAGCTCATTTGGAC-3′; U6, forward, 5′-CTCGCTTCGGCAGCACA-3′, reverse, 5′-AACGCTTCACGAATTTGCGT-3′; TGIF2, forward, 5′-AGAGTGCACTGCATGATAGCGTTCT-3′, reverse, 5′-CCAATGATAAAACAACCATTTGG-3′; GAPDH, forward, 5′-GTCGATGGCTAGTCGTAGCATCGAT-3′, reverse, 5′-TGCTAGCTGGCATGCCCGATCGATC-3′. The PCR amplification reaction was carried out in a 20-μl system, including 1 μl cDNA, as well as 1 μl forward primer and 1 μl reverse primer. The amplification reaction containing 40 cycles was as follows: degeneration for 10 s at 95°C, then followed by reannealing for 20 s at 58°C and finally extension for 34 s at 72°C. Data processing was conducted by 2^−ΔΔ*C*_t_^ method.

### Luciferase reporter assay

Target Scan was used to predict the targetted relationship between *miR-34* and TGIF2, and 3′-UTR was the binding site of *miR-34* and TGIF2. The wild- or mutant-type 3′-UTR of TGIF2 was inserted into the pcDNA3.1/HisC vector (Invitrogen, U.S.A.) to transfect MG-63 cells. Then the psiCHECK2 firefly luciferase reporter plasmids as well as *miR-34* mimics or *miR-34* negative control were used to transfect the MG-63 cells by Lipofectamine 2000 (Invitrogen, U.S.A.). According to the difference in transfection type, cells are grouped as follows: MT + mimics group, MT + NC group, WT + mimics group, and WT + NC group. Cells of each group were seeded in 24-well plates at a density of 1 × 10^5^/ml and 1 ml cell suspension was added into each well. Then these 24-well plates were incubated in 5% CO_2_, 37°C, 95% humidity carbon dioxide incubator. After 48 h of incubation, these cells were collected and luciferase activity was performed by dual-luciferase reporter assay system according to the manufacturer’s protocol (Promega, U.S.A.).

### Establishment of osteosarcoma nude mice model

Twenty-five male nude mice (aged 5–6 weeks) without statistical differences in body weight were housed under aseptic conditions. Water and feed were also sterilized. After 1 week of feeding, all nude mice were underwent skin disinfection. Then a total of 1-ml cell suspension (with a density of 1 × 10^4^/ml) of each group was injected subcutaneously into the right dorsal limb. Cell suspension of each group was injected with five nude mice. These nude mice were also divided into blank group, *miR-34* mimics group, NC group, TGIF2 group, and TGIF2 + mimics group based on the difference of injected cell suspension. After injection, these nude mice were returned to the cage and kept for 6 weeks. At 1, 2, 3, 4, 5, and 6 weeks of injection, long diameter (a) and short diameter (b) of subcutaneous tumors were measured using a Vernier caliper. Tumor volume was calculated by the following formula: tumor volume = (a × b^2^)/2. Six weeks after injection, all nude mice were anesthetized and subcutaneous tumor was removed. Part of each tumor was paraffin-embedded to prepare tissue sections for subsequent immunohistochemistry and immunofluorescence detection. The remaining part of each tumor was without any treatment and used for Western blot and apoptosis researches. Animal studies have been approved by our ethics committee.

### Western blot

Total proteins of each tumor tissues were extracted by using RIPA lysis buffer. Then these proteins were separated through SDS/PAGE before being transferred on to the PVDF membrane. Skimmed milk at a concentration of 5% was used to block the membrane for 2 h incubation. The membrane was placed in an incubator and mouse anti-human TGIF2 monoclonal antibody (1:1000, purchased from Cw Biotech, Shanghai, China) was added for incubation at 4°C overnight. The membrane was washed by TBST for three times with 10 min each time. Goat anti-mouse secondary antibody (1:5000, purchased from Beijing Zhong Shan Biotechnology Co., Ltd., China) was served as secondary antibody for 1 h of incubation. Again, three times washing by TBST was conducted. At last, ECL reagents were used to detect blotted protein. GAPDH was set as internal reference in this research.

### Immunofluorescence detection

Tumor tissue sections were incubated for 15 min at room temperature with 0.25% Triton X-100, followed by being blocked with 4% goat serum for 30 min. Then TGIF2 antibody (1:100) was added for 12-h incubation at 4°C. After washing by PBS for three times, rhodamine labeled fluorescent secondary antibody (1:200) was added for additional incubation of 40 min in an incubator at 37°C. Fifteen minutes of DAPI staining was performed and cells were observed under fluorescence microscope. The number of TGIF2-positive cells was counted.

### Apoptosis detection by flow cytometry

Osteosarcoma tissues were used to detect cell apoptosis by flow cytometry. A 120-mesh stainless steel mesh was placed in a small beaker. Osteosarcoma tissues of each group were cut into small pieces and placed on the 120-mesh stainless steel mesh. These small tissue pieces were gently rubbed using eye tweezers accompanied by flushing with saline. Then the cell suspension was collected and centrifuged at 1000 rpm. Ethidium Bromide (50 μg/ml) and RNaseA (100 μg/ml) were added to these cells for 30-min incubation at 4°C in darkness. At last, flow cytometry was used to detect apoptosis.

### Immunohistochemistry to detect caspase-3 expression

Five consecutive sections of each tumor tissue were selected and were deparaffinized in xylene. After rehydration by a series of graded alcohols, 0.01 M sodium citrate (pH 6.0) was used to perform antigen retrieval. Then these tumor tissue sections were blocked by goat serum for 15 min at room temperature. Primary antibody was added for 12-h incubation at 4°C, followed by secondary antibody for 15 min incubation at 37°C. Total 40 μl of horseradish enzyme-labeled streptavidin solution was used for 15-min incubation at 37°C after washing by PBS for three times. At last, DAB color reaction was carried out and Hematoxylin was used for counterstaining for 30 s. Five slices of each section were randomly selected to count caspase-3 positive cells and percentage of positive cells was calculated. Cells with brown particles in cytoplasm were considered as caspase-3 positive cells.

### Statistical analysis

Data were analyzed using SPSS 18.0 statistical software and was presented as means ± S.D. The comparison between two different groups was performed by *t*test and differences were considered statistically significant if *P*<0.05.

## Results

### Down-regulation of *miR-34* in osteosarcoma tissues and cells

*miR-34* expression in tumor tissues and non-tumor tissues of patients with osteosarcoma was determined by qRT-PCR. The results showed that *miR-34* relative expression in tumor tissues was significantly lower than that in non-tumor tissues (*P*<0.05) (Figure 1A). In addition, *miR-34* relative expression, prominently decreased, was also found in MG-63 cells compared with that in hFOB 1.19 cells (*P*<0.05) (Figure 1B).

**Figure 1:** *miR-34* expression by qRT-PCR (**A**) *miR-34* expression in tumor tissues and non-tumor tissues of patients with osteosarcoma by qRT-PCR; (**B**) *miR-34* expression in hFOB 1.19 cells and MG-63 cells by qRT-PCR. *P<0.05.

### *miR-34* inhibited growth and promoted apoptosis of osteosarcoma in nude mice

Amongst blank group, NC group, and *miR-34* mimics group, *miR-34* relative expression in *miR-34* mimics group was obviously higher than that in the other two groups (*P*<0.05). Meanwhile, no significant difference was found between blank group and NC group (Figure 2A). Up-regulation of *miR-34* expression was successfully achieved by transfection.

**Figure 2:** *miR-34* inhibited osteosarcoma growth and promoted its apoptosis in nude mice (**A**) *miR-34* expression of tumor tissues in each group nude mice by qRT-PCR; (**B**) tumor volume of nude mice in each group; (**C**) apoptosis of tumor tissues in each group nude mice by flow cytometry; (**D**) caspase-3 expression by immunohistochemistry. *P<0.05 when compared with blank group or NC group, respectively.

Nude mice *in vivo* transplantation experiment results showed that, during 4–6 weeks, the tumor volume of *miR-34* mimics group was significantly lower than that of blank group and NC group (*P*<0.05). From 1 to 6 weeks, there was no significant difference in tumor volume between blank group and NC group (Figure 2B). Flow cytometry showed that the percentage of apoptotic cells in *miR-34* mimics group was much higher than that in blank group and NC group (*P*<0.05) (Figure 2C). This result was also confirmed by immunohistochemistry that caspase-3 positive cells proportion of *miR-34* mimics group was markedly higher than that of blank group and NC group (*P*<0.05) (Figure 2D). Above results suggested that up-regulation of *miR-34* inhibited osteosarcoma growth and promoted its apoptosis in nude mice.

### *miR-34* regulated TGIF2 expression targetly

According to Western blot, TGIF2 protein relative expression of tumor tissues of nude mice in *miR-34* mimics group was dramatically lower than that in blank group and NC group (*P*<0.05) (Figure 3A). Immunofluorescence detection also showed that the proportion of TGIF2 positive cells of tumor tissues of nude mice in *miR-34* mimics group was significantly lower than that in blank group and NC group (*P*<0.05) (Figure 3B). These results illustrated that *miR-34* had an impact on the expression of TGIF2.

**Figure 3:** *miR-34* regulated TGIF2 expression targetly (**A**) TGIF2 protein expression of tumor tissues in each group nude mice by Western blot; (**B**) TGIF2 positive cells proportion of tumor tissues in each group nude mice by immunofluorescence; (**C**) prediction of binding sites between TGIF2 and *miR-34* by TargetScan; (**D**) dual luciferase reporter assay. *P<0.05 when compared with blank group or NC group, respectively.^ #^*P*<0.05 when compared with blank group or NC group, respectively.

We further researched the above speculation with TargetScan, and found that 3′-UTR region was the binding site of TGIF2 to *miR-34* (Figure 3C). To verify this result, luciferase reporter experiments were then performed. As a result, no statistically significant difference was found in luciferase activity between MT + mimics group and MT + NC group. However, dramatically lower luciferase activity was presented in WT + mimics group compared with that in WT + NC group (*P*<0.05) (Figure 3D), which indicated that *miR-34* could targetly regulate TGIF2 expression.

### *miR-34* inhibited growth and promoted apoptosis of osteosarcoma in nude mice through targetting regulated TGIF2 expression

Further studies were conducted to investigate the mechanism of *miR-34* in inhibiting growth and promoting apoptosis of osteosarcoma in nude mice. For tumor tissues of blank group, TGIF2 group, and TGIF2 + mimics group, *TGIF2* mRNA and protein relative expression was significantly higher than than of blank group (*P*<0.05), while no statistically significant difference was observed between TGIF2 + mimics group and blank group in *TGIF2* mRNA and protein relative expression (Figure 4A,B).

**Figure 4:** *miR-34* inhibited growth and promoted apoptosis of osteosarcoma in nude mice through targetting regulated TGIF2 expression (**A**) *TGIF2* mRNA expression of tumor tissues in each group nude mice by qRT-PCR; (**B**) TGIF2 protein expression of tumor tissues in each group nude mice by Western blot; (**C**) tumor volume of nude mice in each group; (**D**) apoptosis of tumor tissues in each group nude mice by flow cytometry; (**E**) caspase-3 expression by immunohistochemistry. *P<0.05 when compared with blank group.

In addition, during 1–3 weeks, there was no statistically significant difference in tumor volume amongst blank group, TGIF2 group, and TGIF2 + mimics group. At weeks 4, 5, and 6, significantly higher tumor volume was found in TGIF2 group compared with that in blank group (*P*<0.05). However, the tumor volume of TGIF2 + mimics group was still not statistically different from that of blank group (Figure 4C).

Meanwhile, flow cytometry results show that, compared with blank group, the percentage of apoptotic cells in TGIF2 group was significantly decreased (*P*<0.05). However, the difference of apoptotic cells percentage between TGIF2 + mimics group and blank group was not statistically significant (Figure 4D). The results of immunohistochemistry also showed that, the proportion of caspase-3 positive cells in TGIF2 group was significantly lower than that in blank group (*P*<0.05), while no significant difference was found between TGIF2 + mimics group and blank group (Figure 4E). All the above results indicated that *miR-34* inhibited growth and promoted apoptosis of osteosarcoma in nude mice through targetting regulated TGIF2 expression.

## Discussion

Osteosarcoma, one of the major malignant tumors, results in relatively higher mortality around the world, especially amongst adolescents and young adults [15–17]. Surgical resection combined with radiotherapy or chemotherapy is the traditional treatment for tumors currently [18,19]. However, patients are often accompanied by a high rate of recurrence [20]. As a common primary sarcoma of bone, the occurrence and development of osteosarcoma have been reported to be related to the abnormal expression of many genes [21]. Several articles have demonstrated that miRNAs play an important role in the development of tumors, which provides an important guideline and theoretical basis for the treatment of tumors at the genetic level [22]. In this paper, *in vivo* studies in nude mice were performed to research the effect of *miR-34* on osteosarcoma growth and apoptosis, and related mechanism was also further studied. The results illustrated that the expression of *miR-34* in osteosarcoma tumor tissues was dramatically down-regulated. The results also revealed that the mechanism of *miR-34* inhibiting growth and promoting apoptosis of osteosarcoma in nude mice was through targetly regulating the expression of TGIF2. To our knowledge, researches about the effects as well as mechanism of *miR-34* on osteosarcoma development were very limited. Our study suggested that *miR-34* might be used as a potential biomarker for osteosarcoma, which provided an important guiding significance for the treatment of osteosarcoma at the molecular level.

*miR-34* was reported to be declined in a variety of tumors, which was recommended as a tumor suppressor miRNA [23–25]. Garofalo et al. [26] researched that *miR-34* was down-regulated in lung tumors. They also found that decreased non-small-cell lung cancer cell migration and invasion could be achieved by *miR-34* overexpression or by down-regulation of PDGFR-α/β. Based on this, their further research identified the relationship between *miR-34* and PDGFR-α/β that PDGFR-α/β was targetly regulated by *miR-34*, which provided a therapeutic target for the treatment of non-small-cell lung cancer. Zhang et al. [27] explored the effect of *miR-34* on the prognosis of patients with gastric cancer. Their results revealed that significant down-regulation of *miR-34* occurred in tumor tissues compared with that in adjacent normal tissues. They also concluded that lymph node metastasis, advanced TNM stage, poor tumor differentiation, as well as high recurrence rate and poor overall survival, was markedly associated with low *miR-34*a expression level. They recommended *miR-34* to be used as a prognostic marker for patients with gastric cancer. Our results were consistent with these previous studies that *miR-34* was down-regulated in osteosarcoma tissues and cells. In addition, we further observed that TGIF2 was the target gene of *miR-34*, and the effect of *miR-34* on inhibiting growth and promoting apoptosis of osteosarcoma was through targetly regulating TGIF2 expression. TGIF2 was reported to be associated with a variety of cancers, whose overexpression significantly promoted the progression or development of many tumors, such as skin cancer, breast cancer [28,29]. Lu et al. [30] showed that inhibition of growth and metastasis of non-small-cell lung cancer cell by *miR-541-3p* could be reversed by TGIF2. Several studies also explored the relationship between miR-34 and TGIF2 in regulating tumor development. Yang et al. [31] revealed that *miR-34a* was dramatically decreased in gastric cancer tissues when compared with that in adjacent non-tumor tissues. They also suggested that up-regulation of *miR-34* could play an inhibitory effect on gastric tumor metastasis and invasion by targetly suppression the expression of TGIF2. In this research, we also found a similar mechanism that *miR-34* could inhibit growth and promoting apoptosis of osteosarcoma by targetly regulating the expression of TGIF2.

In conclusion, this article researched the effect of *miR-34* on osteosarcoma and the results showed that *miR-34* was down-regulated in osteosarcoma. More importantly, *miR-34* inhibited growth and promoted apoptosis of osteosarcoma through targetly regulating the expression of TGIF2. It was of significant importance for the treatment of osteosarcoma in clinical at molecular level.

## Abbreviations

DMEM: dulbeccos modified eagle medium
FBS: fetal bovine serum
GAPDH: glyceraldehyde-3-phosphate dehydrogenase
MT: mutant-type
NC: negative control
PDGFR-α/β: platelet-derived growth factor receptor-α/β
qRT-PCR: real-time quantitative reverse transcription polymerase chain reaction
RIPA: radio immunoprecipitation assay
TGIF2: transforming growth factor-β-induced factor homeobox 2
TNM: tumor node metastasis
WT: wild-type
